RETRACTED

# The Value of Rivaroxaban Combined with Ticagrelor in Antithrombotic Therapy after PCI in Patients with Nonvalvular Atrial Fibrillation with Acute Coronary Syndrome

**DOI:** 10.1155/2022/4807175

**Published:** 2022-11-03

**Authors:** Zhengwang Liu, Xiaotang Qiu, Hua Yang, Xiaocui Wu, Wenjing Ye, Xinbing Zheng

**Affiliations:** ^1^Department of Cardiovascular Medicine, Chinese Traditional Medicine Hospital of Hainan Province, Haikou, Hainan 570203, China; ^2^Department of Endocrinology, Hainan Hospital of Traditional Chinese Medicine, Haikou, Hainan 570203, China; ^3^Clinical Research Center of Hainan Provincial Hospital of Traditional Chinese Medicine, Haikou, China

## Abstract

**Objective:**

Based on a retrospective cohort study, to investigate the value of rivaroxaban combined with ticagrelor in antithrombotic therapy after PCI in patients with nonvalvular atrial fibrillation with acute coronary syndrome.

**Methods:**

A total of 60 patients from January 2019 to May 2021 accepted therapy with antithrombotic therapy after PCI. The patients treated with ticagrelor were set as the control group, and those given rivaroxaban combined with ticagrelor were set as the research group. The curative effect, myocardial level, TIMI blood flow grade, platelet aggregation rate, and the incidence of cardiovascular events were taken from the comparisons.

**Results:**

The research group's therapeutic impact was superior to the control group's therapeutic impact, and the value was higher. After treatment, the myocardial levels of the two groups decreased, and the levels of troponin I, creatine kinase isoenzyme, and hypersensitive C-reactive protein in the research group were greatly less than those in the control group, and the difference was statistically significant (*P* < 0.05). After operation, the TIMI blood flow classification in the experimental group was better than that in the control group, and the difference was statistically significant (*P* < 0.05). The experimental group's platelet aggregation incidence was considerably lower than the control group's platelet aggregation incidence at 0.5 and 2 hours following surgery, and the difference was statistically significant (*P* < 0.05). The incidence of acute myocardial infarction, cardiogenic death, and intractable angina pectoris in the research group was significantly lower than that in the control group.

**Conclusion:**

Rivaroxaban combined with ticagrelor in the treatment of nonvalvular atrial fibrillation with acute coronary syndrome after percutaneous coronary intervention; the TIMI blood flow grade is better than ticagrelor, which is of great significance to reduce mortality and has high safety in clinical application.

RETRACTED

## 1. Introduction

Coronary heart disease (CHD) has gradually become one of the most important disorders threatening lives [1]. Acute coronary syndrome (ACS) is a common cardiovascular disease in clinical practice. For these kinds of patients, acute treatment requires revascularization, and follow-up treatment requires antiplatelet therapy. Patients with ACS need to take antiplatelet drugs for a long time to decrease the occurrence of acute coronary ischemic events, especially for patients after percutaneous coronary intervention (PCI) in order to prevent in-stent thrombosis and recurrent myocardial ischemic events.

Patients with nonvalvular atrial fibrillation complicated with acute coronary syndrome often need anticoagulation therapy for atrial fibrillation to reduce the incidence of circulatory embolism. Antiplatelet therapy is usually a combination of antiplatelet therapy (DAPT), in which aspirin is combined with a P2Y12 receptor inhibitor (clopidogrel, prasugrel, ticagrelor) [2], which is the basis for the prevention of coronary ischemic events after acute coronary syndrome or percutaneous coronary intervention. Clopidogrel is the most studied P2Y12 receptor inhibitor. The combination of clopidogrel can reduce the incidence of cardiovascular death. The Tseng Andrew et al. [3] study demonstrated that although the rate of massive bleeding increased by 38% in the entire cohort after using clopidogrel for 1 year, the benefits of clopidogrel outweighed the risk of bleeding, which had nothing to do with patient management and revascularization strategies (PCI or coronary artery bypass grafting). However, many pharmacodynamic studies have consistently shown that individuals have different responses to clopidogrel and there is interindividual and intraindividual variability [4]. Ticagrelor can effectively inhibit the reuptake of adenosine by balanced nucleoside transporter-1 (ENT-1) on the surface of red blood cells, which further strengthens the local adenosine reaction, thus achieving additional inhibition of platelet aggregation and activation and has a good protective effect on vasodilation and myocardial tissue [5]. Because of its above advantages, it has been recommended by a number of relevant guidelines around the world to be used in the antiplatelet treatment of acute coronary syndrome so that more patients can benefit from it [6].

At the same time, more and more evidence showed that the recurrence of atherosclerotic thrombosis, including stent thrombosis and recurrent myocardial infarction, may be attributed to the resistance of some patients to clopidogrel, which is closely related to CYP2C19 gene polymorphism. Clopidogrel's irreversible blockade of adenosine diphosphate (ADP) receptor P2Y12 on platelets has become a vital factor in acute coronary syndrome because it can significantly improve the prognosis. However, there are three disadvantages to the application of clopidogrel (delayed action, irreversible platelet inhibition, and susceptibility to genetic polymorphism of cytochrome P-450 isozymes). The responsiveness of patients to clopidogrel varies a lot from one person to the next. Based on the above reasons, other drugs have been developed, such as new platelet P2Y12 inhibitors, which have a stronger inhibitory effect on platelets than clopidogrel. The use of new platelet P2Y12 inhibitors (prasugrel, ticagrelor) in patients treated with PCI has been widely proven to improve the clinical prognosis of patients [7]. Ticagrelor is a new type of oral antiplatelet drug called cyclo-pentyl-triazolyl pyrimidine (CPTP). Its chemical structure is obviously different from that of thiophene pyridines such as clopidogrel (clopidogrel) and prasugrel (prasugrel). After entering patients with acute coronary syndrome, the drug can exert its effect and take effect quickly without liver metabolic activation, and can rapidly bind to P2Y12 adenosine diphosphate receptor and play the role of antiplatelet over aggregation [8].

RETRACTED

Patients are often complicated with atrial fibrillation, resulting in a significant increase in the risk of adverse events, so anticoagulation therapy for atrial fibrillation is often needed to reduce the incidence of circulatory embolism. Compared with the traditional oral anticoagulant warfarin, the new oral anticoagulants (NOACs) have the advantages of rapid action, no food interaction, less drug interaction, and predictable pharmacokinetics [9]. It is gradually being widely used in clinical practice, especially the use of rivaroxaban, which increased from 0.13% to 13.87% from 2011 to 2014 [10]. Rivaroxaban is accepted to prevent stroke, systemic embolism, and thrombosis after hip and knee arthroplasty. Studies have shown that rivaroxaban is as safe and effective as warfarin [11, 12]. Rivaroxaban has the advantages of rapid action, no food interaction, less drug interaction, and predictable pharmacokinetics. Ticagrelor takes effect quickly after entering patients with acute coronary syndrome, does not need liver metabolic activation, can quickly bind to P2Y12 adenosine diphosphate receptor, plays the role of antiplatelet excessive aggregation, and has a good protective effect on vasodilation and myocardial tissue. Theoretically, the combination of the above two drugs can improve the prognosis of patients. Based on this, a retrospective cohort study was conducted to explore the value of rivaroxaban combined with ticagrelor in antithrombotic therapy after PCI in patients with nonvalvular atrial fibrillation with acute coronary syndrome. The results are as follows.

RETRACTED

## 2. Materials and Methods

### 2.1. General Information

A total of 60 cases with nonvalvular atrial fibrillation with acute coronary syndrome in our hospital from January 2019 to May 2021 were treated with antithrombotic therapy after PCI. The patients treated with ticagrelor were set as the control group, and those treated with rivaroxaban combined with ticagrelor were set as the research group. The control patients' age ranged from 34–74 years old (50.63 ± 3.42), including 18 males and 12 females. The study patients' age ranged from 33 to 76 years (50.73 ± 3.43), including 16 males and 14 females. Our hospital approved by the ethical committee accepted the trial, and all patients signed written permission forms. There was no significant difference in general data between the two groups. This is a retrospective cohort study.

#### 2.1.1. Selection Criteria

Selection criteria were defined as follows: (1) discharge diagnosis of atrial fibrillation, including atrial fibrillation during admission or previous history of atrial fibrillation; all patients meet the diagnostic criteria of atrial fibrillation [11]; (2) admission diagnosis of ACS and secondary PCI; (3) informed consent of the subjects; and (4) age >18 years old.

#### 2.1.2. Exclusion Criteria

Exclusion criteria were defined as follows: (1) rheumatic valvular disease, biological valve, or mechanical valve repair; (2) patients who were hospitalized again after being enrolled in this study; (3) severe underlying diseases such as malignant tumor, blood system diseases, severe liver and renal dysfunction; (4) rheumatic immune system diseases; (5) age <18 years old; and (6) pregnant women.

### 2.2. Methods

The control patients accepted ticagrelor 90 mg/twice a day. In this process, all patients were treated with antimyocardial ischemia therapy (nitrate lipids, angiotensin inhibitors, and receptor blockers) and lipid-regulating and plaque-stabilizing therapy (statins).

The cases of the observation group accepted rivaroxaban, ticagrelor 10 mg/once a day, and ticagrelor tablets (H20193177) 90 mg/twice a day. Patients in both groups took the drug continuously for one year.

### 2.3. Observation Index

#### 2.3.1. Clinical Curative Effect

Refer to the criteria for the evaluation of the efficacy of ACS complicated with atrial fibrillation in the guidelines (2016) [13], which are effective: symptoms such as angina pectoris basically disappear; effective: the clinical symptoms are significantly improved, and the degree of symptoms is reduced by 50%; ineffective: the clinical symptoms are not alleviated or even aggravated. Total effective = effective + effective.

RETRACTED

#### 2.3.2. Myocardial Injury

The fasting venous blood samples were collected, and the levels of troponin I, creatine kinase isoenzyme, and hypersensitive C-reactive protein were detected by table analyzer, rate method, and immunoturbidimetry.

#### 2.3.3. TIMI Blood Flow Classification

The TIMI blood flow classification criteria [14] are as follows: grade 0: coronary artery is completely blocked, no contrast medium passes through; grade 1: contrast medium can penetrate the blocked part but cannot fill the distal coronary artery bed; grade 2: the contrast medium can fill the entire coronary artery, but the blood flow velocity is slower than that of normal vessels and the emptying of the contrast medium is delayed at the distal end of the stenosis. Grade 3: the contrast medium completely filled the whole coronary artery, and the flow rate was consistent with that of normal blood vessels, and the contrast medium emptying was normal [15].

#### 2.3.4. Platelet Aggregation Rate

The platelet aggregation rate was measured by the turbidimetric method before PCI, 0.5 h and 2 h after taking the drug. Within 2 hours, the professionals in the laboratory department used the PRECILLBY-NJ four-channel platelet aggregator to detect platelet aggregation rate, and 10 mol/L adenosine diphosphate was used as inducer.

#### 2.3.5. Cardiovascular Events

Cardiovascular events (MACE) include acute myocardial infarction, cardiogenic death, and intractable angina pectoris.

### 2.4. Statistical Analysis

SPSS23.0 statistical software was adopted to process the data. The measurement data were presented as ($\bar{x}$ ± *s*). The group design *t*-test was adopted for the comparison, and the analysis of variance was adopted for the comparison between multiple groups. The Dun-net-t test was adopted for comparison with the control group. The counting data were presented in the number of cases and the percentage, *χ*^2^ test was adopted for comparison between groups, and bilateral test was employed for all statistical tests.

## 3. Results

### 3.1. Comparison of Curative Effect

In comparison of the curative effect, the research group had an efficiency of 96.67%; the normal group had an efficiency of 73.33%. The research curative effect was greater than that of the control group, and the difference was statistically significant (*P* < 0.05). All the results are shown in Figure 1.

### 3.2. Comparison of Myocardial Level

After drug therapies, the myocardial level was found to decrease. The research group's troponin I, creatine kinase isoenzyme, and hypersensitive C-reactive protein showed less in comparison with the control group, and the difference was statistically significant (*P* < 0.05).  Table 1 depicts just about all the collected data.

RETRACTED

### 3.3. TIMI Blood Flow Grading Comparison

Compared immediately after operation, the interventional group's TIMI blood circulation categorization was greater than the control group's, the findings were statistically meaningful, and the difference was statistically significant (*P* < 0.05).  Table 2 depicts just about all the collected data.

### 3.4. Comparison of Platelet Aggregation Rate

The platelet aggregation rate at 0.5 h and 2 h after operation in the observations was significantly lower than that in the control group, and the difference was statistically significant (*P* < 0.05).  Table 3 depicts just about all the collected data.

### 3.5. The Incidence of Cardiovascular Events 30 Days after Operation

The research incidence of acute myocardial infarction, cardiogenic death, and intractable angina pectoris was significantly lower than that in the control group, and the difference was statistically significant (*P* < 0.05). All the results are shown in Figure 2.

## 4. Discussion

Atrial Fibrillation (AF) occurs with a frequency of 1%, 2%, and 0.5% in subjects aged 40–50 years old. The reported prevalence in adults over the age of 80 ranges from 5% to 15% [16]. According to the Global Burden of Disease Study published in 2014, it is estimated that more than 20 million men and 12 million women worldwide suffer from atrial fibrillation, with nearly 5 million new cases of atrial fibrillation each year [17]. Based on our prevalence model and US census data and 2050 projections, we estimate that the number of cases of atrial fibrillation may increase threefold over the next 50 years, of which 35%, 43%, and 22% are attributable to increased morbidity, population aging, and population size, respectively [18]. Atrial fibrillation is a type of supraventricular arrhythmia, which is characterized by disordered atrial activation and subsequent deterioration of atrial mechanical function, which makes the heart lose its normal systolic and diastolic function, which is conducive to the formation of atrial thrombosis. Shedding leads to strokes and other system embolism [19, 20]. In addition, the loss of synchronization between the atrium and the ventricle leads to atrial and ventricular mechanical dysfunction, followed by heart failure and dysfunction. Compared with patients with sinus rhythm, patients have impaired life quality, decreased cognitive function, and increased mortality. Atrial fibrillation brings a great mental and economic burden to patients and society. Existing clinical evidence shows that standard anticoagulation therapy can decrease embolic events and enhance the prognosis of patients [21]. A retrospective cohort study was conducted to explore the value of rivaroxaban combined with ticagrelor in antithrombotic therapy after PCI in patients with nonvalvular atrial fibrillation with acute coronary syndrome.

RETRACTED

In clinical practice, acute coronary syndrome, especially after PCI treatment, is more closely related to atrial fibrillation. For these patients, atrial fibrillation is considered to be the reason for death. Explanations of potential mechanisms include disappearance of atrial contraction, decreased atrioventricular synchrony, increased filling pressure, enhanced cardiac remodeling, deterioration of left ventricular systolic dysfunction, increased incidence of ventricular arrhythmias, and sudden cardiac death [22, 23], in which the proportion of patients complicated with ACS is high and the prognosis is poor. So far, the exact mechanism of new atrial fibrillation in patients with acute coronary syndrome is not clear, which may be related to atrial ischemia or atrial infarction, inflammatory reaction, changes in autonomic nervous tension, increased atrial pressure, and so on. Whether it is new-onset atrial fibrillation or previously defined atrial fibrillation, the risk of long-term death is also significantly increased. Previous research implied acute coronary syndrome could increase the risk of atrial fibrillation by 2.3% to 37%, resulting in a five-fold increase in in-hospital mortality [24]. Greene's study shows that about 6 to 8 percent are associated with atrial fibrillation or other diseases that require oral anticoagulants, and 20 to 30 percent also have ischemic heart disease [25]. According to the new AHA/ACC/HRS guidelines in 2019, the proportion accounts for 10–21%, that is, 1-2 out of every 10 patients are complicated with atrial fibrillation. Although in recent decades we have observed a decrease in the probability, which is probably linked to the early patency of diseased blood vessels and the widespread use of related drugs, such as *β*-blockers, ACEI/ARB, and aldosterone receptor antagonists [26], the disease burden caused by acute coronary syndrome with atrial fibrillation cannot be ignored.

ACS patients tend to have atrial fibrillation. Once atrial fibrillation occurs, the ejection fraction of the heart will be greatly reduced. At the same time, it will increase the risk of mural thrombosis and its disability and mortality. Several reports have found that among AF patients over 65 years old, 1/3 of patients are complicated with coronary heart disease [27]. In addition, atrial fibrillation has a higher risk of heart failure, thromboembolic events, and hospitalization [28]. Therefore, we need to strengthen the treatment for acute coronary syndrome. Oral anticoagulants can reduce the risk of stroke and systemic embolism [29]. The effects of the two cannot be replaced by each other, but the combination of these two kinds of drugs increases the risk of bleeding, so how to find the balance of antithrombotic therapy in these patients is very important, and the risk of bleeding and thrombus needs to be fully assessed to maximize the benefit of patients.

RETRACTED

Rivaroxaban is a selective inhibitor of Xa factor, which can inhibit free and bound coagulation factor Xa and prothrombin activity [30], thus exerting an anticoagulant effect [31]. Ticagrelor is the first fully synthetic drug developed by AstraZeneca for acute coronary syndrome, including drug therapy and percutaneous coronary intervention. It is also the first reversible oral P2Y12 adenosine diphosphate receptor antagonist [32]. The chemical structure of the drug is cyclo-pentyltriazole pyrimidine, which acts directly on the P2Y12 receptor through intestinal absorption, reversibly binds to it, and then plays a strong antiplatelet effect. At present, ticagrelor has been completed in pharmacokinetic studies in healthy people, patients with acute coronary syndrome [33], and patients with atherosclerosis. The mean plasma concentrations of ticagrelor parent drug and active metabolites, as well as the time to peak and the drug dose, showed a significant linear correlation, which is important for stable coronary atherosclerosis. It is especially important for patients with sclerosing heart disease and atherosclerosis. In the pharmacodynamic study, the inhibition rate of platelet aggregation (IPA) of ticagrelor at a loading dose of 180 mg was significantly higher than that of clopidogrel at a loading dose of 600 mg. The inhibition of platelet aggregation was detected at any time point after 24 hours of administration. Even in the maintenance phase, ticagrelor at 90 mg/time, twice a day is still higher than clopidogrel at 75 mg/time, once a day [34]. This is consistent with the idea recommended in the guidelines of the European Heart Association and the American Heart Association as an alternative to ticagrelor. With the widespread use of clopidogrel in clinical practice, clopidogrel resistance generally occurs and shows a further upward trend in the study of individual differences. Platelet aggregation cannot be fully inhibited under clopidogrel resistance [35]. On the other hand, ticagrelor has a good effect on antiplatelet aggregation and it can also exert a good effect on platelet inhibition in patients with acute coronary syndrome who are resistant to clopidogrel. The platelet aggregation rate decreased from (59 ± 9) (%) to (35 ± 11) (%), especially 24 hours after percutaneous coronary stent implantation. The ideal antiplatelet effect can be obtained by using ticagrelor in patients with clopidogrel resistance or acute coronary syndrome with low response [36]. In addition, the pharmacodynamic activity of ticagrelor was not affected by the liver CYP2C19 gene polymorphism. At present, gene polymorphism is the main reason that affects the variability of clopidogrel response, which makes the antiplatelet effect of the drug difficult to predict, coupled with the widespread existence of CYP2C19*∗*2 alleles in the population, which brings uncertainty to its therapeutic effect. This study has some limitations: the sample size of this study is small, it belongs to a single-center study, and there is a certain deviation. There are patients' own factors and other confounding factors that may interfere with the accuracy of this study. In future research, we will carry out multicenter, large-sample prospective studies, from which we can draw more valuable conclusions.

RETRACTED

To sum up, when rivaroxaban is combined with ticagrelor in the treatment of nonvalvular atrial fibrillation with acute coronary syndrome after percutaneous coronary intervention, the TIMI blood flow grade is better than ticagrelor, which is of great significance to reduce mortality and has high safety in clinical application.

## Figures and Tables

**Figure 1:** Comparison of curative effect between the two groups.

**Figure 2:** Comparison of cardiovascular events 30 days after operation between the two groups.

**Table 1:** Comparison of myocardial level between the two groups ($\bar{x}\pm s$).

Grouping	*N*	Troponin I level (Ng/L)		Creatine kinase isoenzyme (U/L)		Hypersensitive C-reactive protein (mg/L)	
		Before treatment	After treatment	Before treatment	After treatment	Before treatment	After treatment
Control group	30	1.89 ± 0.33	1.35 ± 0.44	18.29 ± 5.33	15.69 ± 2.56	8.93 ± 1.42	7.84 ± 0.69
Research group	30	1.83 ± 0.31	1.02 ± 0.33	18.20 ± 5.31	13.45 ± 2.31	8.99 ± 1.65	6.33 ± 1.33
*t* value		0.725	3.286	0.065	3.558	0.150	5.519
*P* value		>0.05	<0.05	>0.05	<0.05	>0.05	<0.05

**Table 2:** Comparison of TIMI blood flow classification between the two groups (*n*/%).

Grouping	*N*	0 stage		1 stage		2 stage		3 stage	
		Before operation	After surgery	Before operation	After surgery	Before operation	After surgery	Before operation	After surgery
Control group	30	21 (70.00)	0	9 (30.00)	0	0	6 (20.00)	0	24 (80.00)
Research group	30	20 (66.67)	0	8 (26.67)	0	0	3 (10.00)	0	29 (96.67)
*t* value		0.077	—	0.082	—	—	1.176	—	4.043
*P* value		>0.05	>0.05	>0.05	>0.05	>0.05	>0.05	>0.05	<0.05

RETRACTED

**Table 3:** Comparison of platelet aggregation rate between the two groups ($\bar{x}\pm s$, (%)).

Grouping	*N*	Before operation	After operation 0.5 h	After operation 2 h
Control group	30	58.93 ± 3.31	40.95 ± 1.45	33.54 ± 1.42
Research group	30	58.39 ± 3.65	33.21 ± 1.35	25.49 ± 1.54
*t* value		0.600	21.398	21.048
*P* value		>0.05	<0.05	<0.05

## Data Availability

The datasets used and analyzed during the current study are available from the corresponding author upon reasonable request.
